The article "Long-Term Assessment of Rehabilitation Treatment of Sports through Artificial Intelligence Research" was published in 2021. Journal: Comput Math Methods Med.

# Long-Term Assessment of Rehabilitation Treatment of Sports through Artificial Intelligence Research

**DOI:** 10.1155/2021/4980718

**Published:** 2021-12-22

**Authors:** Chaofan Zeng, Ying Huang, Longer Yu, Qingmei Zeng, Bijun Wang, Yi Xu

**Affiliations:** ^1^Guangzhou Institute of Technology, Guangzhou, Guangdong 510075, China; ^2^Guangdong Foreign Trade School, Guangzhou, Guangdong 510520, China; ^3^Rehabilitation Department, The Fifth Affiliated Hospital, Southern Medical University, Guangzhou 510900, China; ^4^Guangdong Eco-Engineering Polytechnic, Guangzhou, Guangdong 510520, China

## Abstract

**Background:**

Artificial intelligence (AI) technology has been incorporated into all walks of life, especially the integration of machine learning and health management has achieved very significant progress and results. It is very necessary to analyze personalized sports health management services and long-term assessment of health issues in the era of AI.

**Methods:**

This paper explores AI + personalized sports management service system design ideas, system operation process, management stage design, taking common chronic diseases, and diabetes as examples. 150 patients were divided into an observation group and a control group, and the blood glucose, blood pressure, blood lipid, and knowledge awareness rate were compared.

**Results:**

The blood glucose, blood pressure, and blood lipid levels of the observation group all reduced, and the awareness rate of diabetes knowledge increased, which proved that the AI research has great value in sports rehabilitation research coupled with long term health assessment and is worth further research.

**Conclusion:**

The AI research proposed in this paper is of far-reaching practical significance in helping the transformation and upgrading of the sports health management service industry, promoting the innovative development of sports health management service supply, and promoting national fitness and national health.

## 1. Introduction

In the past 20 years, population aging, cancer rejuvenation, and subhealth have become the focus of public health concerns [1]. The elderly have been suffering from osteoporosis and cardiovascular and cerebrovascular diseases for a long time. Lymphoma, gastric cancer, and other cancer patients are more common in young and middle-aged people, and most of them are found in the middle and late stages, and the mortality rate increases year by year. The distribution of China's population health status shows that only 5% are healthy people and 80% are subhealthy people, of which about 300 million are obese people [2, 3].

Long-term subhealth causes chronic diseases. The number of deaths caused by chronic diseases has accounted for 86% of the total deaths in the country 6%, and the burden of chronic diseases accounts for nearly 70% of the total disease burden. Chronic diseases have become a health crisis that people cannot ignore.

In 2018, China entered the first year of AI and became a new generation of AI innovation development test area. Nearly 30 provinces, cities, and regions issued relevant planning documents or issued supporting policies to promote the development of the AI industry. AI leaders, benchmarking companies, and specialized small and medium-sized enterprises produce a series of smart products with different functions such as sports wearable smart devices, online health management services, and real-time monitoring of health data. Residents can use these smart products to monitor and understand their own health status, help residents self-health information query function and exercise monitoring, evaluation, promotion, and provide personalized health management services for residents [4–7].

China's sports health management service already has AI products and technology penetration, but it is not deep enough. The theoretical research on the application of AI in sports health management services is still very weak, and social development is in urgent need of sports health management services. Therefore, the research on the design of personalized sports health management service system in the era of AI will help the transformation and upgrade of sports health management service industry. To promote the innovative development of sports health management services, promote national fitness and national health, and provide a reference for the healthy development of China.

Personalized sports health management is a process of comprehensive monitoring, analysis, evaluation, and management of residents' physical health [8]. Through effective personalized sports fitness guidance and behavioral intervention, the purpose of improving residents' health levels and self-health management capabilities is achieved, thereby a new sports service process that promotes the health of athletes [9].

## 2. Methodology

### 2.1. AI + Personalized Sports Management Services

#### 2.1.1. System Design Ideas

As can be seen from Figure 1, based on the sports health management service monitoring-evaluation-intervention-promotion, the AI + personalized sports health management service system is constructed. The four service links of health information management system, sports health assessment management, fitness guidance and intervention, and sports health promotion use AI equipment or technology to achieve fast, convenient, and scientific fitness management.

First, wearable smart products are used to monitor the true and reliable health data of residents, and a sports health cloud information system is established; then, residents and sports managers collect personal or group monitoring health cloud data and initially diagnose the health status of residents or groups through APP software or smart instruments and conduct sports health assessment to build sports health assessment management; then, individual residents or groups use scientific sports fitness projects, methods, or means to conduct fitness guidance and behavior intervention strategies in smart fitness venues.

Finally, residents can use the online knowledge base or interactive communication between sports health managers, to obtain feedback information for self-health management, to achieve health promotion. In order to build an AI sports health management service system, the entire system design idea not only helps residents' self-health information query function and exercise monitoring, evaluation, and promotion but also facilitates sports health managers to use intelligent platform data more flexibly, targeting different ages and different groups of people, individuals, or groups of different ranges customize personalized physical and health exercise programs.

We build a sports health management service system and use the sports health cloud management system to act on community sports health management services, athlete sports health management services, corporate sports health management services, sports health management services for the elderly, pregnancy and health management services, youth sports health management services, chronic disease sports health management services, physical health management services in eight areas, provide AI technology sports guidance, and form a series of health management service systems. A series of health management service systems have been continuously improved and improved, and on the contrary, the efficiency of sports health management service links has been promoted.

#### 2.1.2. System Operation Flow

As can be seen from Figure 2, the operation process of the AI + personalized sports management service system is relatively complicated and cumbersome. The system subverts the traditional sports health management model, builds a new sports health management system of the Internet of Things and cloud computing, and adopts a vertical structure layered and horizontal cross-domain, vertical layered to complete the real-time health data recording of fitness people, information transmission, file collection, storage, calculation, processing, and security of collected data, to achieve the formation of various application programs and user reports on data and information transformation. Horizontal cross-domain interconnection, sharing, and collaborative processing with various clouds truly realizing the dynamic multidimensional management of national sports health records throughout the life cycle, providing sports health managers with dynamic data of health records, and providing real-time sports for users or residents health management services provides online sports service platforms for sports health instructors.

#### 2.1.3. Management Stage Design

From Figure 3, the sports health management service link is divided into six links: sports health information collection system, sports health status assessment and prediction, sports health management plan formulation, sports health intervention, sports health promotion, and sports health evaluation; the size is included in the systematic management stage, the refined management stage, and the individualized management stage; according to the different work priorities, the sports and health managers who undertake the above work can be divided into social sports instructors, fitness management consultants, and personal trainers.

Residents then communicate, maintain, promote, and improve sports health management through the network with sports managers. Healthy residents or subhealthy residents can all self-monitor, self-control, self-discover problems, and self-analyze problems through intelligent software or network platforms. In the form of self-seeking solutions, when residents find that the exercise effect is not obvious, they can consult with online sports managers in time to obtain the most favorable fitness prescription. All of this can be done through AI software or instruments, bringing great convenience to residents, enhancing residents' knowledge and ability of active sports health management, saving time and effort, and bringing scientific and technological progress to the application of AI technology to the field of sports.

### 2.2. Implementation Path of Long-Term Sports Health Management Services in the Era of AI

#### 2.2.1. Implementation Path of Self-Help Sports Health Service in the Unit of Family or Hospital

As can be seen from Figure 4, the self-service sports health service in the family unit is a resident health management information platform built by a third-party health operation organization, which provides remote sports health management information operation services for family members, forming a self-service sports fitness management service application based on family places system and application system of physical therapy and fitness management service with hospital as a place.

The family self-help sports health service application platform is a sports health information operation service organization that provides family members with sports prescriptions, technical guidance and consultation, and other information services. Provide self-service health online services to family members through mobile sports APP applications, WeChat, websites, or smart devices, including health file services, sports consulting services, sports fitness services, sports fitness assessment and guidance, and sports effect evaluation.

The physical therapy fitness management service application platform takes the hospital as a place, performs reasonable and effective rehabilitation physical therapy for the sick, and combines medical and physical therapy to build a physical medicine management contact service station. Specific operation steps establish an electronic medical record database, combine the online fitness guidance platform with medical treatment, provide fitness guidance and help needs, and provide people with online professional fitness coaches in a timely and effective manner to guide people in fitness exercises and improve the accuracy of guidance and efficiency and formulate effective exercise prescriptions.

In the process of sports rehabilitation, through the medical evaluation service, the changes in the disease can be evaluated to avoid physical damage caused by improper exercise. And to determine whether sports services are beneficial to patients' health and disease recovery, so that sports services can timely adjust exercise programs, assessment, and promotion processes according to patients' own diseases or health conditions.

#### 2.2.2. The Implementation Path of Sports Health Management Services in Athletes

It can be seen from Figure 5 that under the unified leadership of the athlete, the sports health management service uses the intelligent equipment or instruments to carry out sports health testing, sports classroom teaching, extracurricular sports activities, sports training, and competition as the main content of the health management system. The specific tasks of athletes' sports health management: health information collection-student sports health management files-student sports health management information analysis and evaluation-personalized sports health guidance, intervention-re-collection-re-evaluation-re-guidance, and intervention management model. That is to pass first collect and manage students' health information through smart software or the Internet and establish student electronic health management accounts and files. The athlete carries out health education and carries out health education on nutrition knowledge, sports fitness knowledge, and sports safety knowledge related to physical health through elective courses, networks, lectures, and reports. Then evaluate the students' health status, formulate fitness and health management programs in physical education classrooms, extracurricular sports activities, sports training, and competitions, and intervene and guide the students' health status.

#### 2.2.3. Implementation Path of Personalized Sports Health Management Services in the Community

Under the leadership of the city and municipal people's government, community sports health management services are led by the streets, and the neighborhood committees are coordinated to establish a sports health management team as a guide to carry out physical fitness tests and sports health events for community residents. Health education system with sports health skills transmission and sports health knowledge dissemination as the main content.

Specific tasks of community sports health management: mainly establish and improve the electronic health files of residents under the jurisdiction of the community health service center and regularly update the data of dynamic changes, which is not only convenient for statistical analysis of data but also convenient for community sports instructors and communities. Medical staff and community residents log in to view the health information of community residents. Second, for community residents, health records are entered into the community sports online health management system. To some extent, the community sports online health management system is a kind of basic public sports and health service with public welfare. For community sports instructors and community medical staff, the entry of health records into the community sports online health management system is conducive to their effective monitoring of health-risk groups.

### 2.3. Value of AI Research on Sports Rehabilitation Research

#### 2.3.1. General Materials

This study selected 130 diabetic patients, divided into two groups according to the random number method, the observation group was given health management, and the control group was given general management, 75 cases each. In the observation group, there were 37 males and 38 females; the average age was (61.25 ± 2.85) years, with an age range of 54 to 72 years; the average course value was (6.02 ± 0.35) years, and the course of disease was 7 months to 12 years. In the control group, there were 38 males and 37 females; the average age was (61.28 ± 2.87) years old, with an age range of 55-72 years; the average course value was (6.06 ± 0.37) years, and the course of disease ranged from 8 months to 12 years.

#### 2.3.2. Comparative Experimental Methods

Control method: give general management, that is, inform patients to take medicines according to doctor's orders and develop good living habits, moderate exercise, etc.

Observation group method: give health management for 6 months, as follows:

1. *Establish a Health Management Team*. The main members are composed of nurses, and doctors and head nurses provide corresponding guidance. Participating members are trained in diabetes-related knowledge and can only be employed if they have passed the training
2. *Investigating the Health Status*. The nursing staff should collect the patient's health information (awareness of the disease, lifestyle, medication, psychological status, etc.), then assess the health risk factors based on the collected information, and then be the inspected person formulate an individualized intervention plan
3. *Health Management Methods*. Nursing staff can carry out health management by regularly conducting health lectures, distributing relevant knowledge manuals, establishing WeChat groups, monthly telephone calls, or follow-up visits
4. *Health Management Content*. (a) Health education: choose appropriate language according to the patient's cultural level to explain disease-related knowledge, such as pathogenesis, inducing factors, clinical manifestations, complications manifestations, and preventive measures and then let them understand and improve recognition knowledge has a significant promoting effect, and then inform patients that diabetes is a lifelong disease. Any treatment method cannot cure the disease. Only drugs can be used to control blood sugar levels, which, in turn, reduce the harm to physical functions, which is conducive to improving the patient's medication. Compliance and develop good habits. (b) Reasonable diet: make reasonable adjustments according to the patient's diet and focus on low-calorie, low-cholesterol, low-fat, low-salt, low-sugar, high-quality protein, and high-fiber, and abide by the principle of a small number of meals. (c) Exercise guidance: inform patients to exercise at least 5 times a week, mainly aerobic exercise, such as brisk walking, yoga, and square dance, can reduce the body weight while improving immunity, at the same time, it can further improve the insulin sensitivity. It is necessary to pay attention to the combination of work and rest during exercise, observe the step-by-step principle, and exercise intensity should be tolerated. (d) Take medicine according to the doctor's instructions: once again emphasize to the patient the importance and necessity of taking the medicine on time and on demand, which is conducive to controlling the disease and preventing the occurrence of complications, and at the same time, explaining the medicine-related knowledge to the patient, such as the method of taking, dosage, and effect, in turn, it plays a role in raising awareness; in addition, it is forbidden to change drugs and increase or decrease the dose of drugs at will

#### 2.3.3. Observation Indicators

Observation and evaluation of systolic blood pressure, diastolic blood pressure, fasting blood glucose, 2 h postprandial blood glucose, glycated hemoglobin, total cholesterol (TC), triglyceride (TG), low-density lipoprotein (LDL-C), high-density lipoprotein (HDL-C), blood sugar, blood pressure, blood lipid, and knowledge awareness rate.

The knowledge awareness rate selection questionnaire is evaluated. The evaluation content includes 6 questions such as pathogenesis, clinical manifestations, etiology, treatment, and complications. It is designed as 25 multiple choice questions, each question has 5 options, and each option score is 0 to 4 points, the total score is 0 to 100 points; of which 80 to 100 points indicate complete awareness, 60 to 79 points indicate partial awareness, and less than 60 points indicate no awareness; the format of knowledge awareness rate is as follows.

(1) $$\begin{array}{c} \text{Awareness rate}=\frac{\text{Fully aware}+\text{Partially aware}}{\text{Total number of cases}}. \end{array}$$

## 3. Results

### 3.1. Comparison of Blood Pressure Levels

The data in Table 1 shows that before intervention, and there was no statistically significant difference in systolic and diastolic blood pressure between the observation group and the control group (*P* > 0.05); after intervention, the systolic and diastolic blood pressure of the observation group was lower than that of the control group, and there was a statistical difference Academic significance (*P* < 0.05). It shows that AI has research value in the rehabilitation treatment of diabetes and can reduce systolic and diastolic blood pressure.

### 3.2. Comparative Analysis of Blood Sugar Levels

The data in Table 2 shows that before the intervention, there was no statistically significant difference between the observation group and the control group's fasting blood glucose, 2 h postprandial blood glucose, and glycated hemoglobin (*P* > 0.05); after intervention, the observation group's fasting blood glucose, postprandial 2 h blood glucose, and glycated hemoglobin were lower than those in the control group, and the difference was statistically significant (*P* < 0.05). In the observation group receiving AI health management, blood glucose levels have decreased significantly.

### 3.3. Comparative Analysis of Blood Lipid Levels

The data in Table 3 shows that before intervention, there was no significant difference in TC, TG, LDL-C, and HDL-C between the observation group and the control group (*P* > 0.05); after intervention, TC, TG, and LDL-C are lower than the control group, HDL-C is lower than the control group, and the difference is statistically significant (*P* < 0.05).

### 3.4. Comparative Analysis of Blood Sugar, Blood Pressure, Blood Lipids, and Knowledge Awareness Rate

The data in Table 4 shows that the observation awareness rate is higher than that in the control group, and the difference is statistically significant (*P* < 0.05). The observation group is receiving AI health management on diabetes pathogenesis, clinical manifestations, etiology, treatment, and complications.

## 4. Discussion

Diabetes is one of the more common chronic diseases in the clinic, with a high morbidity rate [10]. If it is not effectively treated in time, it can have a serious impact on the health of the patient. At present, there is no complete cure for the disease in the clinic, only by taking drugs to play a role in controlling the disease and have a positive effect on reducing the incidence of complications [11]. However, due to the low awareness of disease-related knowledge in some patients, it is easy to cause repeated fluctuations in blood glucose levels, and the predisposing factors are poor eating habits and lifestyle habits. (1) Have not taken medicine according to doctor's instructions. Some scholars have shown that good metabolic control for diabetic patients is conducive to avoiding the appearance of chronic complications and has a significant promoting effect on life extension. Therefore, it is very important to find suitable intervention methods in the clinic [12].

Smart technology has been applied to nearly 20 industries such as shopping malls, hotels, banks, museums, hospitals, and teaching and will be used in various fields of society in the future [13].

At present, wearable smart devices such as smart bracelets, smart sports shoes, smart glasses, and smart shirts in the sports and fitness industry have become indispensable sports products for residents' fitness. It can monitor user's health data in real time and timely feedback on sports effects, so that residents can know your own health status accurately [14, 15]. Deep learning can be used for automatic diagnosis of the patient in future [16–19]. China has used the intelligent physical fitness test system to complete the student's physical fitness test files, exercise risk prediction, scientific new fitness training, and fitness effect monitoring and other technical means to provide basis and services for the prevention, intervention, and improvement of athlete's health. The APP software is used to monitor the pace, calories, cadence, heart rate, etc. in real time during the fitness exercise and make the most suitable exercise intensity fitness management service plan in time. These intelligent products will inevitably lead the sports health management service to personalization and provide convenient conditions to meet individual needs.

## 5. Conclusion

Through AI, we can effectively study the value of sports rehabilitation research. After investigation, it is found that diabetes is a metabolic disease, not only the phenomenon of elevated blood sugar but also abnormal performance of blood pressure and blood lipids. Therefore, it is necessary to implement a long-term health management of patients clinically to achieve control of blood sugar levels and improve blood pressure and blood lipids. Health management is mainly carried out from the aspects of education, diet, sports, and medical treatment. The premise is to establish a management team, through the training of group members, to improve the comprehensive quality of nursing staff, and then better the provision of services by patients has a positive effect on improving the quality of care and patient satisfaction.

## Figures and Tables

**Figure 1:** Design framework of AI + personalized sports management service system.

**Figure 2:** Operation flow chart of AI + personalized sports management service system.

**Figure 3:** Design diagram of AI + personalized sports health service management stage.

**Figure 4:** Roadmap for the implementation of self-service sports and health services by families.

**Figure 5:** Implementation road map of athletes sports health service management.

**Table 1:** Comparison of blood pressure levels of the two patients.

Group	Number of cases	Systolic blood pressure		Diastolic blood pressure	
		Before intervention	After intervention	Before intervention	After intervention
Observation group	75	146.47 ± 10.46	125 ± 5.24	92.44 ± 4.67	80.24 ± 1.03
Contrast group	75	145.64 ± 10.27	129 ± 6.75	94.21 ± 4.35	87.55 ± 2.77
*t* value	—	0.021	7.012	0.024	21.471
*P* value	—	0.991	0.001	0.936	0.001

**Table 2:** Comparison of blood glucose levels of the two patients.

Group	Fasting blood glucose (mmol/L)		2 h blood glucose after meal (mmol/L)		Glycated hemoglobin (%)	
	Before intervention	After intervention	Before intervention	After intervention	Before intervention	After intervention
Observation group (*n* = 75)	10.68 ± 3.11	8.66 ± 0.99	14.21 ± 3.46	7.46 ± 1.52	9.11 ± 2.03	6.31 ± 0.67
Contrast group (*n* = 75)	9.96 ± 2.86	7.46 ± 1.02	13.19 ± 2.76	8.76 ± 1.98	9.31 ± 1.33	6.96 ± 0.77
*t* value	0.072	7.786	0.012	5.963	0.068	13.256
*P* value	0.939	0.001	0.943	0.001	0.996	0.001

**Table 3:** Comparison of blood lipid levels between the two patients.

Group	TC		TG		LDL-C		HDL-C	
	Before intervention	After intervention	Before intervention	After intervention	Before intervention	After intervention	Before intervention	After intervention
Observation group (*n* = 75)	4.75 ± 1.33	2.33 ± 0.34	1.86 ± 0.68	0.96 ± 0.03	2.78 ± 0.75	1.67 ± 0.16	1.24 ± 0.68	2.04 ± 0.89
Contrast group (*n* = 75)	4.86 ± 0.68	7.46 ± 1.02	1.55 ± 0.65	1.26 ± 0.36	2.33 ± 0.64	2.19 ± 0.52	1.35 ± 0.86	1.46 ± 0.85
*t* value	0.195	14.468	0.194	4.671	0.167	14.003	0.427	4.613
*P* value	0.855	0.001	0.821	0.001	0.864	0.001	0.876	0.001

**Table 4:** Comparison of blood glucose, blood pressure, blood lipid, and knowledge awareness levels of the two patients.

Group	Number of cases	Fully aware	Partially aware	Do not know	Awareness rate (%)
Observation group	75	56	17	2	97.33
Contrast group	75	50	14	11	85.33
*X* ^2^ value	—	—	—	—	7.134
*P* value	—	—	—	—	0.007

## Data Availability

The image data used to support the findings of this study have been deposited in the diabetes dataset (https://www.kaggle.com/naveenkhasa/pima-indian-diabetes-dataset).
